# The molecular fingerprint of lung inflammation after blunt chest trauma

**DOI:** 10.1186/s40001-015-0164-y

**Published:** 2015-08-25

**Authors:** Christian Ehrnthaller, Michael Flierl, Mario Perl, Stephanie Denk, Heike Unnewehr, Peter A. Ward, Peter Radermacher, Anita Ignatius, Florian Gebhard, Arul Chinnaiyan, Markus Huber-Lang

**Affiliations:** Department of Traumatology, Hand-, Plastic-, and Reconstructive Surgery, Center of Surgery, University of Ulm, Albert-Einstein-Allee 23, 89081 Ulm, Germany; Department of Orthopaedic Surgery, School of Medicine, University of Colorado, Aurora, USA; Department of Pathology, University of Michigan, Ann Arbor, USA; Anesthesiological Pathophysiology and Process Development, University of Ulm, Ulm, Germany; Institute of Orthopedic Research and Biomechanics, Center of Musculoskeletal Research, University of Ulm, Ulm, Germany; Michigan Center for Translational Pathology, Universtiy of Michigan, Ann Arbor, USA; BG-Trauma Center Murnau, Murnau, Germany

**Keywords:** Blunt chest trauma, Inflammation, Microarray, Transcription program

## Abstract

**Background:**

After severe blunt chest trauma, the development of an acute lung injury (ALI) is often associated with severe or even lethal complications. Especially in multiple injured patients after blunt chest trauma ALI/ARDS [acute respiratory distress syndrome (ARDS)] is frequent. However, in the initial posttraumatic phase, inflammatory clinical signs are often not apparent and underlying changes in gene-expression profile are unknown.

**Methods:**

Therefore, inflammation in lung tissue following blunt chest trauma was characterized in a well-defined bilateral lung injury model. Using DNA microarrays representing 9240 genes, the temporal sequence of blunt chest trauma-induced gene-expression patterns in lung tissue was examined.

**Results:**

The results suggest an activation of a highly complex transcriptional program in response to chest trauma. Chest trauma led to elevated expression levels of inflammatory and coagulatory proteins (such as TNFα receptor, IL-1α, IL-1β, C3, NF-κB and plasminogen activator). However, upregulation of proteins was found, usually incoherent of exerting effects in blunt thoracic trauma (pendrin, resistin, metallothionein and glucocorticoid-induced leucine zipper). Furthermore, significant downregulation was observed as early as 10 min after trauma for cytokines and complement factors (LCR-1, C4) as well as for intracellular signaling molecules (inhibitory protein phosphatase) and ion-channels (voltage-dependent Ca^2+^ channel).

**Conclusions:**

Taken together, the provided global perspective of the inflammatory response following blunt chest trauma could provide a molecular framework for future research in trauma pathophysiology.

## Background

Severe trauma to the chest with pulmonary contusion still causes approximately a quarter of all civil trauma-related deaths [1]. Especially for lung injury inflicted by blasts (e.g. in the crime/military setting), the underlying pathophysiology and development of the inflammatory response is still poorly understood [2]. Various biological mediators seem to play a central role in the pathophysiology of blunt chest trauma, including cytokines, complement (e.g. C5a) and coagulation factors [3]. Persistent elevation of pro-inflammatory cytokines in the lungs with subsequent suppression (or increasing paralysis) of the immune system is associated with an enhanced risk for acute lung injury (ALI) progression and is known to increase mortality. We have previously demonstrated, that lung contusion is the major contributor to posttraumatic inflammation even in combined injury and in the presence of hemorrhagic shock, suggesting that the degree of pulmonary inflammation is an important determinant for the clinical course post-trauma [4]. Many cytokines and other pro-inflammatory mediators, such as complement activation products, involved in the development and progression of ALI are known to be regulated via the transcriptional regulatory factor nuclear factor (NF)-κB. Yet, ALI is a highly complex poly-etiological syndrome, which cannot only be triggered by various local damage (such as lung contusion, blunt chest trauma, pneumonia or ventilatory damage to the lung [2]), but it may also be triggered by limited remote injury (such as long bone fractures, head trauma) and also by different systemic insults such as large volume blood transfusions, burn injuries, shock, polytrauma [5], systemic inflammatory response syndrome (SIRS) and sepsis. However, the underlying changes in protein expression profiles are rather speculative. Therefore, in the present study, we used a 9240 element rat cDNA microarray to analyze pulmonary gene-expression patterns in a well-characterized rat model of blunt chest trauma [6]. Various pro-inflammatory mediators are currently routinely measured in plasma in the face of a very dynamic and rapidly changing environment in trauma to assess the “trauma load” and serve as predictive markers for the patient´s course and outcome [7]. In contrast, data from and extrapolations to individual organs are hardly achievable in the clinical setting. Based on our blunt chest trauma model, microarray analysis of pulmonary gene expression may provide important insights into the pulmonary pathophysiology after blunt chest trauma, which might ultimately help to mitigate or, perhaps, prevent the progression to ALI/ARDS. Furthermore, the present findings identify potential new candidates and facilitate prediction of the clinical outcome supporting the development of new therapeutic strategies.

## Methods

### Animals and anesthesia

All investigative procedures and the animal facilities conformed with the Guide of Care and Use of Laboratory Animals published by the US National Institutes of Health. The study was approved by the regional animal care and use committee (Approval No. 784/2003). Adult pathogenic-free male Wistar rats (325–375 g, Charles River, Wilmington, MA, USA), were anesthetized with a mixture of 2.5 % sevoflurane (Sevorane TM Abbott, Wiesbaden, Germany) and 97.5 % oxygen (under continuous flow of 3 l/min). The gas combination was applied by a mask covering the snout of the animal. To continue adequate analgesia after injury, buprenorphine (0.03 mg per kg body weight) was injected subcutaneously every 6 h. Before and after surgery, rats had unrestricted access to food and water.

### Blast-induced bilateral lung injury

Blunt chest trauma was induced on anesthetized rats by a single blast wave centered on the thorax as previously described [6]. In surviving animals, no extrathoracic injuries (such as liver rupture etc.) were found macro- and microscopically. The upper section of the device served as a pressure reservoir and was separated from the lower nozzle by a 50 µm Mylar TM polyester film (Du Pont, Bad Homburg, Germany). The pressure reservoir was connected to a storage tank of compressed air. Between both components an electronically releasable high-speed valve (Hee-D-24, FESTO, Esslingen, Germany) and a pressure reducing valve set to 13 bar (Zinser, Ebersbach, Germany) were interposed. By opening the high-speed valve, compressed air was delivered into the upper section of the generator. When the pressure exceeded the resistance of the polyester diaphragm, the film ruptured towards the nozzle, releasing a well-defined single blast wave. The nozzle-chest-distance was strictly kept at 2 cm, leading to acute mortality rates of about 5 % (immediate cardiac rupture, posttraumatic apnea). Each blast wave was highly reproducible as assessed by a pressure transducer (Omega 100 psi, New Port Omega, Dechenpfronn, Germany) attached horizontally to the opening of the nozzle. Sham-treated animals were equally anesthetized and received equal volumes of PBS. The following time-points were investigated post-trauma: sham, 10 min, 1, 3, 6, 12 and 24 h. All time points and different treatment groups (sham, blunt chest trauma) consisted of *n* = 5–7 per experimental condition.

### Isolation of mRNA

At given time-points after trauma, lungs were flushed with 10 ml PBS to remove blood cells. Total RNA was extracted from lungs using Trizol reagent (Life Technologies, Grand Island, NY, USA) according to the manufacturer’s instructions and stored at −80 °C until further analysis. Control mRNA samples were isolated from sham animal lungs.

### Microarray analysis

DNA microarray analysis of gene expression was done as described at [8] and by the Brown and Derisi Labs (available at http://www.microarray.org). The sequence-verified cDNA clones of the rat cDNA microarray are available from Research Genetics (http://www.resgen.com). Purified polymerase chain reaction products, generated using the clone inserts as template, were spotted onto poly-l-lysine-coated microscope slides using an Omnigrid robotic arrayer (GeneMachines Inc., San Carlos, CA, USA) equipped with quill-type pins (Majer Precision Engineering, Tempe, AZ, USA). One full print run generated ~100 DNA microarrays. All chips have various control elements, which include human, rat, and yeast genomic DNAs, standard saline citrate, yeast genes, housekeeping genes, among others. In addition, we have separately obtained ~500 inflammation- and apoptosis-related cDNAs from Research Genetics to serve as independent controls for clone tracking and function as duplicates for quality control. Protocols for printing and postprocessing of arrays are available in the public domain (http://www.microarray.org). Once isolated, mRNA from both experimental and control organs were used as a template for cDNA generation using reverse transcriptase. Inclusion of amino allyl-dUTP in the reverse transcriptase reaction allowed for subsequent fluorescent labeling of cDNA using monofunctional *N*-hydroxy succinimidyl (NHS) ester dyes (as described [8]). The experimental cDNA sample was coupled to a monofunctional Cy5-NHS ester and the reference cDNA sample to a Cy3-NHS ester (Amersham, Arlington Heights, IL, USA). The labeled probes were then hybridized to 8K rat cDNA microarrays. Fluorescent images of hybridized microarrays were obtained using a GenePix 4000A microarray scanner (Axon Instruments, CA, USA).

### Data analysis

Primary analysis was done using the Genepix software package. Images of scanned microarrays were gridded and linked to a gene print list. Initially, data were viewed as a scatter plot of Cy3 versus Cy5 intensities. Cy3 to Cy5 ratios were determined for the individual genes along with various other quality control parameters (e.g. intensity over local background). The genepix software analysis package flags spots as absent based on spot characteristics (http://www.moleculardevices.com). Additionally, bad spots or areas of the array with obvious defects were manually flagged. Spots with small diameters (<50 µm) and spots with low signal strengths <350 fluorescence intensity units over local background in the more intense channel were discarded. Flagged spots were not included in subsequent analyses. Data were scaled such that the average median ratio values for all spots were normalized to 1.0 (done separately for each array). An arbitrary cut-off ratio of twofold was used to select genes as significantly up- or down-regulated relative to the control sample. Normalized fluorescence ratios of non-flagged array elements were uploaded to a Microsoft Access Database (Microsoft Corporation, Redmond, WA, USA). The data were log2 transformed and hierarchically clustered with average linkage clustering and visualized using the TreeView program. In some cases, inclusion thresholds were increased to focus the returned clusters.

### Protein assays

All protein assays were analyzed using a commercially available ELISA kit in accordance with the manufacturer’s protocol (heme-oxygenase 1; ADI-EKS-810A; Enzo Life Sciences Inc, NY 11735, USA) (Metallothionein; E-EL-R0629; Elabscience Biotechnology Co. Ltd., Wuhan, China) (Resistin; Fa. DRG Instruments Gmbh, Marburg, Germany).

### Statistical analysis

All values of the microarray experiment were expressed as mean ± SEM. Animal groups were individually queried for genes that were differentially expressed in the trauma lungs as compared to negative control lungs. Gene expression was considered statistically significant when trauma group/control ratio was >2.0 (upregulation) or <0.5 (downregulation). For statistical evaluation of the protein analysis an unpaired *t* test (IBM SPSS Statistics 20.0, SPSS Inc., IBM, Armonk, NY, USA) was assessed after testing of normal distribution. Results with *p* ≤ 0.05 were considered statistically significant.

## Results and discussion

### Results

To facilitate access to the high numbers of screened genes, microarray findings were sorted into groups of different mediator systems, cascades and pathways known to be involved in inflammation.

### Cytokines/chemokines

In line with evidence from the literature, transcriptional programs of pro-inflammatory cytokines/chemokines and/or their corresponding receptors were found to be upregulated during the course after blunt chest trauma (Fig. 1). Gene expression for IL-1α was found to be upregulated about threefold very early after trauma (1 h) while expression of IL-1β reached significant upregulation after 12 h and persisted until 24 h. The genes for the TNFα-receptor (TNFα-R) displayed a robust upregulation 1 h through 6 h after blunt chest injury. It was found that chest trauma also seemed to decrease gene-expression levels of some pro-inflammatory cytokines and chemokines with a significant decrease of the chemokine receptor LCR-1 at 1 and 12 h after trauma (Fig. 1).

**Fig. 1:** Regulated genes encoding for various cytokines or their receptors at different time-points after blunt chest trauma. Upregulation was defined as >2-fold increase of gene expression, while downregulation was considered significant when expression levels <0.5 when being compared to sham lungs. *LCR-1* leucocyte chemokine receptor, *TNFα* tumor necrosis factor α. Displayed are mean values ± SEM

### Intracellular pathways

Trauma-induced transcriptional alterations of selected molecules involved in intracellular signaling are exhibited in Fig. 2. As early as 1 h after trauma, the G-protein coupled receptor protein reached a significant upregulation (up to threefold; Fig. 2). MAPK-6 remained significantly elevated from 1 h until 6 h post-trauma. Over the full observation period, there were various intracellular signaling molecules whose genomic expression was diminished after chest trauma (Fig. 2). E.g., expression of the inhibitory protein phosphatase was reduced 1–24 h after injury. MKP-21 showed significantly decreased levels over the whole observation period whereas for MKP-4 a trend towards elevated levels could be detected (data not shown).

**Fig. 2:** Genes encoding for molecules involved in intracellular signaling following blunt chest trauma. Expression ratio of trauma lungs/sham lungs >2 was defined as upregulation, a ratio of <0.5 as downregulation. *MAPK* mitogen activated protein kinase, *MKP* mitogen activated protein kinase phosphatase. Displayed are mean values ± SEM

### Coagulation system

The coagulation system was one of the first biological cascades to respond to blunt chest trauma. Expression of the genes encoding for the plasminogen activator tissue and plasminogen activator urokinase receptor were significantly increased 1–3 h after exposure to blunt chest trauma (Fig. 3).

**Fig. 3:** Lung gene expression involving proteins from the coagulation system, the NF-κB family, and ion-channels at different time-points after chest trauma. Expression ratio of trauma lungs/sham lungs >2 was defined as upregulation, a ratio <0.5 as downregulation. Displayed are mean values ± SEM

### NF-κB family

One of the transcriptional key factors involved in the inflammation-triggered production of cytokines and chemokines is the nuclear transcription factor (NF)-κB. While gene expression of NF-κB light chain was upregulated as early as 10 min and 1 h post-trauma, the inhibitor (IκB) light chain, which regulates NF-kappa B by distinct mechanisms, did not show significant alterations (Fig. 3).

### Ion-channels

Expression of the voltage-dependent calcium channel was decreased over the whole experimental period after trauma and almost abolished 3 h after trauma (Fig. 3).

The pendrin gene codes for the integral membrane protein SLC26A4 exchanging anions for chloride and is strongly expressed in tissues of the kidney, the inner ear and the thyroid. The expression rate of pendrin constantly rose, reaching significant values after 6 h. In the latter course of trauma, pendrin further rose, reaching its peak 12 h after chest trauma (Fig. 3).

### Complement system

Own previous results described an involvement of the powerful complement anaphylatoxin, C5a, in the pathogenesis of blunt chest trauma [3]. Moreover, we observed significant systemic increases of C3a levels following lung contusion (unpublished data). In accordance with these findings, genomic expression of C3 was very significantly elevated 12 h after trauma (Fig. 4), while expression levels of another complement protein, C4, were little affected after chest trauma (Fig. 4).

**Fig. 4:** Expression changes of components of the complement system demonstrate upregulation of C3 and little change in C4. Expression ratio of trauma lungs/sham lungs >2 was defined as upregulation, a ratio <0.5 as downregulation. Displayed are mean values ± SEM

### Cytoprotective proteins

Various cytoprotective proteins, which have not been previously described in blast-induced blunt chest trauma showed significant alterations in the time-course of blunt chest trauma.

Five-fold upregulation was seen for cytoprotective *heme*-*oxygenase 1 (HO*-*1)*. Heme-oxygenase 1 is a stress-responsive enzyme that catabolizes heme into carbon monoxide (CO), biliverdin and iron, thereby providing antioxidant, anti-apoptotic, anti-inflammatory and immunomodulatory properties. While remaining at normal levels directly after trauma, a robust increase occurred 3 h after trauma, sustained 24 h post-trauma, with the highest elevation 12 h after trauma.

Another gene that revealed enhanced expression rates after trauma was the *glucocorticoid*-*induced leucine zipper (GILZ)*. GILZ mediates glucocorticoid actions, such as binding and inhibiting of NF-κB, modulation of T-lymphocyte activation, interleukin production, apoptosis and cell proliferation. As early as 10 min after trauma, significant upregulation was found, peaking at 1 h after the insult. Upregulation persisted until 6 h post-trauma returning to normal levels after 12 and 24 h (Fig. 5).

**Fig. 5:** Expression changes of specific proteins in the lungs during the time-course of blunt chest trauma. Expression ratio of trauma lungs/sham lungs >2 was defined as upregulation, a ratio <0.5 as downregulation. *HO-1* heme-oxygenase 1, *GILZ* glucocorticoid-induced leucine zipper. Displayed are mean values ± SEM

R*esistin,* only recently described as an adipocyte-specific hormone being related to insulin resistance in obese mice, showed by far the most upregulated expression values. The expression rate for resistin significantly increased 3 h after trauma with maximum levels at 12 h (up to sixfold), decreasing until 24 h after induction of blunt chest trauma.

The group of *metallothionein* protein are metal binding proteins that play a role in metal homeostasis, detoxification and removement of oxygen radicals. Metallothionein 1 expression significantly increased early (1–3 h) after trauma.

### Detailed analysis of HO-1 upregulation

Evaluation of heme-oxygenase 1 showed a strong correlation with the microarray data. Significantly elevated levels of HO-1 were found after 3 (*p* = 0.015), 6 (*p* < 0.001) and 24 h (*p* = 0.038) (Fig. 6), while the result after 12 h lacked significance (*p* = 0.063). Metallothionein 1 also showed increased, but not significantly elevated levels after 10 min (*p* = 0.101) and 6 h (*p* = 0.216) (data not shown). However, for resistin, no differences and no correlation with the massive upregulation in the microrarray analysis was seen.

**Fig. 6:** ELISA-based analysis of heme-oxygenase 1 (HO-1) during the time-course of blunt chest trauma in ng/mg protein. Displayed are mean values ± SEM; *p < 0.05

## Discussion

While blunt chest trauma is a common associated injury in multiple injured patients and is accompanied with high morbidity [1], we are only beginning to understand the pathophysiological changes following blunt lung injury. In the present study, we seek to provide a global perspective of the inflammatory response following blunt chest trauma and present a molecular framework for future research in this area. While the gene expression of inflammatory proteins and members of the coagulation/complement cascade showed expected values, proteins which are currently not the focus of research in blunt chest trauma (especially cytoprotective proteins) showed significantly upregulated levels.

### Cytokines/chemokines

Increased levels of IL-1β and IL-1α have been described to be involved in the pathogenesis of ARDS and subsequent pulmonary fibrosis [9]. In line, IL-1β has been reported to be increased in brochoalveolar lavage (BAL) fluids after blunt chest trauma [10], a result which was could be confirmed (Fig. 1). The generally accepted involvement of TNFα-R in the inflammatory cascade was also found to be upregulated in the present study. Overexpression of TNF-α-R seemed to increase the receptor for the complement activation product C5a (C5aR) and to be crucially involved in recruitment of inflammatory cells, as TNF-α-R-knockout mice displayed a decreased neutrophil rolling and adhesion [11].

### Intracellular pathways

MAPK phosphatases (MKPs) are capable of dephosphorylation of activated MAPKs. This results in inactivation of MAPKs with effective abolishment of their physiological functions. During the last years, MKPs have been shown to be crucially involved in the regulation of immune responses. In this regard, MKPs are able to modulate the production of pro- and anti-inflammatory cytokines, innate immune cell viability, the function of antigen-presenting cells and the adaptive immune responses through regulation of cytokine biosynthesis and cell proliferation. Moreover, MKPs serve as a feedback control mechanism of MAPK pathways [12]. In the present study, the MAPKs were found to be upregulated almost over the whole observation period while MKPs showed ambiguous results with elevated (not significant) levels after 1 h (MKP-4) and diminished amounts over the whole experiment for MKP-21 (Fig. 2). MPKs are known to be induced by hydrogen peroxide [13], which might originate from transmigrated neutrophils and macrophages involved in the inflammatory response following blunt chest trauma. In accordance, MPKs have been described to be massively upregulated in response to hypoxia [14], which has been described to occur in the early phase post-trauma in current model [6]. Moreover, MPKs seems to play a critical role in mediating stress responsiveness and regulating inflammatory response in macrophages [15].

### Coagulation system

One of the very early genomic alterations due to blunt chest trauma are the changes in the coagulation system (Fig. 3). The plasminogen activator urokinase receptor, which was found to be significantly increased 1–3 h after trauma, has been described to be upregulated by IL-1β and TNF-α [16], both of which have been reported to be increased early following clinical and experimental blunt chest trauma [10]. In addition, plasminogen activator has been reported to regulate recruitment of white blood cells via upregulation of integrins such as vascular cell adhesion molecule (VCAM) and intracellular adhesion molecule (ICAM) [17], and seems to be a potent chemoattractant for phagocytes. Finally, increased levels of plasminogen activator have been found to be involved in the pathogenesis of lung fibrosis, a classical feature of late stage ARDS [18].

### NF-κB family

Especially early after trauma (10 min and 1 h), NF-κB light chain was one of the highest upregulated proteins in our microarray within the first 3 h. After 3 h expression levels gradually dropped.

Early elevation of NF-κB is not surprising, as it is known, that NF-κB represents a transcriptional factor binding to promoter regions of pro-inflammatory genes such as IL-1β, IL-6, IL-8 and TNF-α being necessary for the production of these crucial inflammatory cytokines [19]. Interestingly, the NF-κB inhibitor was unaltered after blunt TXT.

### Ion-channels

The main function of pendrin, which was highly regulated after thoracic trauma (TXT), is the exchange of anions for chloride. Pendrin is strongly expressed in tissues of the kidneys, the inner ear and the thyroid gland [20]. In kidneys, pendrin maintains acid–base balance by secreting HCO3^−^ in exchange of Cl^−^. In the inner ear, pendrin is of major importance for the generation of the endolymphatic fluid while in the thyroid gland, pendrin functions as a Cl^−^/I^−^ exchanger for maintaining the iodide efflux into the follicular lumen [20]. It has been shown, that pendrin is upregulated in airway epithelium upon inflammatory stimulation of IL-4, IL-13 or antigen exposure [21]. In the last years, increasing evidence has been found that pendrin is upregulated and may be involved in the pathogenesis of pulmonary diseases like asthma or chronic obstructive pulmonary disease (COPD) [20]. In both clinical entities pendrin has been shown to regulate/increase the viscosity of the airway fluid by its distinct function as anion/chloride exchanger, therefore contributing to asthma and COPD exacerbations [22]. Besides the possible upregulation due to the blunt thoracic trauma as inflammatory stimulus, the pathogenic role for pendrin in this injury model remains to be elucidated.

### Complement system

We found that, C3 was strongly upregulated on a genomic level with small changes in C4 (Figs. 1, 4). The local production of complement component C3 by monocytes appears to be regulated, in part, by IL-1β and INF-γ [23]. It is tempting to speculate that the observed upregulation of C3 in lungs after trauma might have been IL1β-mediated. Moreover, systemic infections like sepsis were found to activate complement, consuming C3 and C4 and generating enhanced levels of C3a and C4a especially in patients succumbing to sepsis [24]. In our study, genomic expression of C4 was downregulated 10 min and 12 h post-trauma (Fig. 4). It may be speculated, that this decrease depicts the downregulation of the classical pathway as for traumatic injuries the main activity of the complement system is generated via the alternative pathway. Interestingly, no alteration of complement factor 5 was found in the microarray analysis. Based on excess of key complement components in the blood (such as C3 and C5), it is noteworthy that posttraumatic anaphylatoxin generation (such as C5a) with subsequent biological consequences may occur without significant trauma-induced alteration of their genetic expression.

### Cytoprotective proteins

Various cytoprotective genes were upregulated as a sign of host protection against exogenous detrimental effects of the blast-induced blunt chest trauma.

A significant increase was seen for *heme*-*oxygenase 1 (HO*-*1*). It has been shown, that HO-1 exerts protective effects in the liver e.g. in transplanted liver grafts as well as after ischemia/reperfusion injuries, spinal cord injuries and in acute kidney injury [25]. To our knowledge, no data exist on the role of HO-1 in experimental blunt chest trauma. While some beneficial effects for HO-1 were found in ALI after experimental sepsis [26], an increase of HO-1 seems to have negative effects on the outcome after acute bacterial infection of the lung in pneumonia-induced sepsis potentially by reducing neutrophil function and host defense [27].

The *glucocorticoid*-*induced leucine zipper (GILZ)* was significantly elevated from 10 min post-trauma until 6 h. GILZ was first discovered in the late 1990s. Extensive studies discovered manifold protein functions, especially modulation of T-lymphocyte activation, interleukin production, apoptosis and cell-proliferation [28]. More recently, besides expression in various tissues, different functions of the GILZ have been described such as involvement in the epithelial Na^2+^ channel (ENaC)-mediated Na^2+^ transport in the kidneys. After glucocorticoid stimulus, upregulation in airway epithelium and mesenchymal stem cells was found [28]. Only recently, GILZ was proposed as an endogenous inflammatory inhibitor in arthritis with potential therapeutic potency [29]. In the traumatic setting of spinal cord injury, GILZ overexpression in T-lymphocytes was proposed to inhibit tissue damage and tissue inflammation [28]. Taken together, GILZ seems to inhibit damage and inflammation in several inflammatory diseases with a new role even in blunt thoracic trauma.

In the present study, *Resistin* exhibited elevated expression levels at 3 h remaining upregulated until the end of the experiment. Whereas in humans resistin is mainly expressed in monocytes, in mice it is also found in adipocytes [30]. Consecutively, alternative functions apart from insulin resistance and diabetes have been described: Resistin inherits a strong pro-inflammatory potential through induction of the cytokine cascade and vice versa induction of resistin by pro-inflammatory cytokines has also been demonstrated. Manifold interactions and possible roles for resistin in the pathogenesis of diseases such as atherosclerosis, rheumatoid arthritis and asthma were shown [31]. Up to now, only little is known about its role in traumatic lung tissue damage. While the exact role of resistin in the majority of involved human pathologies remains unclear, regulation of resistin may be regarded as a potential biomarker for the activity of the disease or the extent of organ dysfunction [32].

The protein *metallothionein*-*1* (MT-1) was significantly elevated 1–3 h after trauma. Besides the main function of metal homeostasis, detoxification and removal of oxygen radicals, further roles include protection against DNA damage and binding/exchange of heavy metals such as zinc, copper and cadmium [33]. While MT-1 and 2 can be detected ubiquitally, expression of MT-3 is limited to the brain and male sexual organs. In contrast to the classical functions of MT-1/2, MT-3 plays its major role in development and programmed apoptosis of brain-cells. In the last years, various studies documented the anti-inflammatory and protective role of metallothionein in tissue trauma. Besides accelerated wound healing, studies demonstrated a protective role of MT in brain tissue and proposed therapeutic potential in neurodegenerative diseases [34]. A protective role in lung tissue was demonstrated by Inoue et al. with levels of MT correlating with the degree of pulmonary inflammation in bacterial- or antigen-related ALI [35]. In summary, upregulation of metallothionein clearly represents a marker for the amount of inflammation after blunt chest trauma and can be regarded as a mechanism of the host to limit tissue damage.

## Conclusions

Taken together, the observed transcriptional alterations in the lungs after blunt chest trauma displayed a strong “yin-yang”-like dualism. While some cytokines (like IL-1α and IL-1β) were found to be upregulated, other members of the chemokine family (LCR-1) were downregulated. Similarly, some components of the complement system exhibited a selective pattern (e.g. C3 and C4). Isoforms of MKPs showed ambiguous results with upregulation of the one and downregulation of the other protein. Similar findings of gene dualism were also reported to be imprinted in the molecular signature of sepsis [8]. Various described proteins (e.g. HO-1, GILZ, resistin) have been first described here to be upregulated during blunt chest trauma-induced lung inflammation.

The main limitation of the study arises from its study design. With a genomic analysis no evidence of an in vivo upregulation on protein level can be made. Therefore, further analysis of the alteration on protein levels of relevant genes should be performed. This was of course assessed by the incorporated ELISA-based analysis of the proteins heme-oxygenase 1, metallothionein and resistin. Sadly, further protein analyses were not possible as commercially available ELISAs for the relevant proteins are scarce for rats. Therefore, future studies should focus on genomic analysis in humans with consecutive protein analysis to extend our knowledge and understanding of blunt chest trauma.

Understanding, on a genomic scale, how an organism responds to severe blunt chest trauma may contribute to an improved clinical outcome and might ultimately put new promising treatment modalities on the horizon.
